# Chronic Eosinophilic Pneumonia in an Adolescent Without Known Risk Factors: A Case Report on a Challenging Lung Disease

**DOI:** 10.7759/cureus.90172

**Published:** 2025-08-15

**Authors:** Joseph O Odeyemi, Leah Nasr, Leah Whitis, Apeksha Sathyaprasad

**Affiliations:** 1 Department of Internal Medicine/Pediatrics, University of Kansas School of Medicine, Wichita, USA; 2 Department of Pediatrics, University of Kansas School of Medicine, Wichita, USA; 3 Department of Pediatric Pulmonology, University of Kansas School of Medicine, Wichita, USA

**Keywords:** alveolar eosinophilia, chronic eosinophilic pneumonia, eosinophilic lung disease, noninfectious pneumonia, pediatric pneumonia

## Abstract

Chronic eosinophilic pneumonia (CEP) is a rare lung disease characterized by eosinophilic infiltration of the lungs. It typically presents with nonspecific respiratory symptoms and can mimic more common conditions such as community-acquired pneumonia (CAP), especially in children, making early diagnosis challenging.

We report the case of a previously healthy 15-year-old girl who presented with a seven-week history of fever, cough, dyspnea, and pleuritic chest pain. Initial treatment for presumed CAP with an inflammatory component, including antibiotics and corticosteroids, provided only transient relief. Persistent symptoms, worsening radiographic findings, and marked peripheral eosinophilia raised concern for an alternative diagnosis. An extensive infectious and autoimmune workup was negative. Bronchoalveolar lavage revealed eosinophilia, and lung biopsy ultimately confirmed CEP. The patient responded dramatically to systemic corticosteroids, with rapid clinical improvement.

This case highlights the diagnostic complexity of CEP in pediatric patients. It underscores the importance of considering eosinophilic lung diseases in cases of recurrent or nonresolving pneumonia, especially when peripheral eosinophilia and characteristic imaging findings are present. Early recognition and treatment with corticosteroids are crucial for a favorable outcome.

## Introduction

Chronic eosinophilic pneumonia (CEP) is a rare idiopathic pulmonary disorder characterized by eosinophilic infiltration of the lung parenchyma [1]. It is more frequently observed in women, nonsmokers, and individuals with a history of atopic conditions or environmental allergen exposure [1]. Certain medications, such as nonsteroidal anti-inflammatory drugs and antibiotics like minocycline and co-trimoxazole, have also been implicated as potential triggers [2]. CEP is estimated to account for less than 3% of all interstitial lung diseases [1].

While the exact pathogenesis remains unclear, CEP is distinguished from acute eosinophilic pneumonia (AEP) by its insidious onset over weeks to months, compared with the rapid onset seen in AEP, which is more strongly associated with smoking and acute environmental exposures [1,3].

Diagnosing CEP can be particularly challenging as symptoms often mimic more common conditions such as community-acquired pneumonia (CAP), and patients may experience transient improvement with corticosteroids, leading to misdiagnosis or delayed workup [3,4]. Additionally, the rarity of the disease contributes to a general lack of awareness among clinicians. Current diagnostic criteria typically require symptoms lasting longer than two weeks, alveolar or blood eosinophilia (>25% eosinophils in bronchoalveolar aspirate or serum eosinophil >1,000/mm^3^), pulmonary infiltrates on chest imaging, and exclusion of other known eosinophilic pneumonia-like allergic bronchopulmonary aspergillosis and parasitic infections [1]. This paper presents a case that underscores the diagnostic complexities of CEP in a previously healthy adolescent patient.

## Case presentation

The patient is a 15-year-old girl with no significant past medical history who was admitted to the hospital in February 2025 after a seven-week history of fever, nonproductive cough, and shortness of breath. She was initially diagnosed with CAP in January 2025, with a chest X-ray showing mixed interstitial and alveolar opacities (Figure 1).

**Figure 1:** Chest X-ray taken in January 2025, showing mixed airspace and interstitial opacities, more pronounced in the peripheral lung fields (yellow arrows)

She was treated with a course of amoxicillin and oral prednisone (40 mg daily for five days), prescribed early by her primary care provider due to the prolonged duration of symptoms and presumed inflammatory component. Only mild and transient symptom improvement was noted. This was followed by treatment with azithromycin and then doxycycline, along with a second five-day course of prednisone, again resulting in only mild but transient symptom relief. Epstein-Barr virus testing ordered by her primary care provider was negative for acute infection.

At the time of her February admission, she reported ongoing shortness of breath and a one-week history of pleuritic chest pain, most prominent in the subcostal area. She continued to experience cough and intermittent fevers, along with almost daily chills and diaphoresis. She also lost 7 pounds between January and February 2025. She denied any recent travel, pet exposure, sick contacts, smoking, vaping, or history of atopy. Initial laboratory values on admission are summarized in Table 1. Notable findings included marked leukocytosis with eosinophilia and thrombocytosis, while her comprehensive metabolic panel was within normal limits.

**Table 1:** Laboratory values on admission

Test	Result	Reference range
White blood cell count	18,100 cells/μL	4,000-11,000 cells/μL
Neutrophils	47%	40-70%
Eosinophils	36%	0-6%
Lymphocytes	13%	20-40%
Hemoglobin	11 g/dL	12-16 g/dL (female)
Platelet count	535,000 cells/μL	150,000-400,000 cells/μL
Comprehensive metabolic panel	Within normal limits	-

Repeat chest X-ray showed worsening of the previously noted mixed airspace opacities, now extensive throughout both lungs, most prominent in the periphery and apices (Figure 2). Additionally, a chest computed tomography scan of the chest revealed extensive consolidative opacities in all five lobes, most prominent in the apices, along with prevascular (1.7 x 1.4 cm) and right hilar (1.3 x 1.0 cm) lymphadenopathy (Figures 3-5).

**Figure 2:** Chest X-ray taken in February 2025, showing worse diffuse mixed airspace opacities bilaterally, more pronounced in in the peripheral lung fields and apices (yellow arrows)

**Figure 3:** Chest CT scan taken in February 2025, showing extensive airspace consolidation bilaterally in the upper lung lobes (red double-headed arrows) CT: computed tomography

**Figure 4:** Chest CT scan taken in February 2025, showing extensive airspace consolidation bilaterally, in the right middle lobe and the left upper lobe (red arrows) CT: computed tomography

**Figure 5:** Chest CT scan taken in February 2025, showing enlarged prevascular lymph nodes (yellow arrows) CT: computed tomography

A comprehensive infectious workup was negative, including blood cultures, histoplasma antigen and antibody testing, aspergillus testing, tuberculosis testing, beta-D-glucan testing, and a respiratory viral panel. She also underwent immunology testing (Table 2), including complement components 3 and 4 (C3 and C4), antinuclear antibody screen, immunoglobulin E, perinuclear anti-neutrophil cytoplasmic antibody, and cytoplasmic antineutrophil cytoplasmic antibody, all of which were within normal limits. Inflammatory markers were elevated while lactate dehydrogenase was within normal limits, and serum uric acid levels were low. The electrocardiogram and transthoracic echocardiogram were grossly unremarkable.

**Table 2:** Summary of immunologic workup p-ANCA: perinuclear antineutrophil cytoplasmic antibody; c-ANCA: cytoplasmic antineutrophil cytoplasmic antibody

Test	Result	Reference range
Complement C3	165 mg/dL	82-167 mg/dL
Complement C4	18 mg/dL	10-34 mg/dL
Immunoglobulin E	231 IU/mL	9-681 IU/mL
p-ANCA	<1:20	<1:20
c-ANCA	<1:20	<1:20
C-reactive protein	75 mg/L	<10 mg/L
Erythrocyte sedimentation rate	75 mm/hour	0-20 mm/hour
Lactate dehydrogenase	169 U/L	140-280 U/L
Serum uric acid	1.8 mg/dL	2.5-7 mg/dL

She subsequently underwent a bronchoscopy with bronchoalveolar lavage (BAL). The BAL fluid was negative on cytology and microbiologic testing, including Gram stain and culture, fungal smear and culture, and *Pneumocystis jirovecii* smear. Notably, the eosinophil count was elevated at 20%. Her symptoms improved briefly during her three-day hospitalization while she was not on any medications, and she was discharged with outpatient follow-up arranged. However, she was readmitted within a week due to worsening chest, rib, and back pain, along with increased shortness of breath. Her white blood cell count on readmission was 21,000 cells/μL, with eosinophils making up 40% of the differential. Other labs remained stable.

She underwent video-assisted thoracoscopic surgery with wedge biopsies from the upper and lower lung lobes. Initial pathology impressions were concerning for pulmonary Langerhans cell histiocytosis, prompting empiric steroid initiation by the pediatric pulmonology team due to dense inflammatory infiltrates consisting of histiocytes, lymphocytes, and eosinophils. She was started on oral prednisone, 30 mg daily.

Final histopathology confirmed fibrinous and organizing eosinophilic pneumonia with scattered multinucleated giant cells, consistent with CEP. Differential diagnoses considered included acute fibrinous organizing pneumonia and pulmonary Langerhans cell histiocytosis, both of which were ultimately ruled out based on histological and clinical findings. After confirmation of the CEP diagnosis, the plan was to continue prednisone 30 mg daily for at least one to two weeks after both clinical symptoms and chest X-ray abnormalities resolved before beginning tapering by 5 mg per month over five to six months.

Following initiation of systemic corticosteroids, the patient showed significant clinical improvement within a few days. At her two-week follow-up, she reported resolution of her chest pain and gradual improvement in respiratory symptoms. However, she developed notable side effects from steroid use, including weight gain, facial puffiness, acne, and mood variability. Due to these concerns, she was continued on steroids with measures in place to manage side effects, while steroid-sparing options such as mepolizumab (Nucala), an anti-interleukin-5 monoclonal antibody, are being considered for her long-term management.

## Discussion

This case highlights the diagnostic challenges of CEP, particularly in pediatric patients, where the condition is exceedingly rare and often not initially considered. The patient's prolonged symptoms, partial and transient response to corticosteroids, and nonspecific imaging findings initially mimicked more common conditions such as CAP. This diagnostic ambiguity, compounded by a negative infectious and autoimmune workup, led to a delayed diagnosis despite progressive clinical deterioration.

A brief comparison with existing literature reveals similarities in presentation and histopathologic features with other pediatric CEP cases, although such reports remain limited [5,6]. Additionally, these reports also highlight the challenges with diagnosing CEP, which are similar to those outlined above. The use of BAL eosinophil count and histopathologic confirmation has been consistently emphasized in reported cases to distinguish CEP from other eosinophilic or interstitial pneumonias [3,7].

Another hallmark of CEP is the peripheral and upper lobe-predominant pulmonary infiltrates, which were evident on this patient’s imaging [8]. However, these radiographic features are not pathognomonic and require integration with clinical and laboratory findings, including eosinophilia and exclusion of other causes. Notably, this case illustrates that BAL eosinophilia may be below the classic diagnostic threshold (>25%), reinforcing the importance of a high index of suspicion and the potential need for tissue biopsy in unresolved cases. Histopathologic confirmation via surgical lung biopsy was essential in establishing the diagnosis in this case, with the final pathology revealing organizing eosinophilic pneumonia, thereby confirming CEP. Prompt initiation of corticosteroid therapy led to rapid clinical improvement, consistent with the well-documented responsiveness of CEP to steroids.

A literature search revealed the absence of a consensus guideline for the diagnosis and management of CEP. The working criteria most often used are the four-point criteria outlined earlier: symptoms lasting longer than two weeks, alveolar or blood eosinophilia, pulmonary infiltrates on chest imaging, and exclusion of other known causes of eosinophilic pneumonia [1]. However, as seen in this case, where BAL eosinophilia was <25%, and as reported in the literature, patients with CEP may lack one or more of these criteria. Although it is well established that patients with CEP respond well to corticosteroids, there is no specific guidance on the optimal dose or duration of therapy. Most clinicians initiate prednisone at 0.5 mg/kg or 30 mg daily and continue for at least two weeks after resolution of symptoms and radiologic abnormalities before beginning the taper [1]. Tapering strategies vary widely, and no regimen has been proven superior. One study found no significant difference in relapse rates between patients tapered over three months and those tapered over six months. Relapses, occurring in up to half of patients, typically respond well to reintroduction of corticosteroids. Biologic agents, including the anti-IgE antibody omalizumab, the anti-IL-5 antibody mepolizumab, and the anti-IL-5 receptor antibody benralizumab, have been used successfully as steroid-sparing maintenance therapy in patients with frequent relapses or steroid intolerance [1]. However, there is no clear guidance on the dosing or duration of these biologics, and most clinicians follow regimens established for other hypereosinophilic syndromes [1].

## Conclusions

CEP is a rare and often underrecognized cause of persistent respiratory symptoms, especially in the pediatric population. This case illustrates the diagnostic challenges posed by its nonspecific presentation, initial partial response to corticosteroids, and overlap with more common conditions like CAP. A high index of suspicion, along with integration of clinical, radiologic, and histopathologic findings, is essential for timely diagnosis. Prompt initiation of corticosteroid therapy can lead to significant clinical improvement, as seen in this patient. This case emphasizes the importance of considering CEP in the differential diagnosis of prolonged pulmonary infiltrates with eosinophilia, even in previously healthy adolescents.
